The article "Protection of rat intestinal epithelial cells from ischemia/reperfusion injury by (D-Ala2, D-Leu5)-enkephalin through inhibition of the MKK7-JNK signaling pathway" was retracted in 2024. Reasons: plagiarism; plagiarized data; overlap with other authors' work; unreliable data.

# Protection of rat intestinal epithelial cells from ischemia/reperfusion injury by (D-Ala2, D-Leu5)-enkephalin through inhibition of the MKK7-JNK signaling pathway

**DOI:** 10.3892/mmr.2015.3991

**Published:** 2015-06-24

**Authors:** ZHENRAN WANG, BO TANG, FANG TANG, YANG LI, GUANGYU ZHANG, LI ZHONG, CHENCHENG DONG, SONGQING HE

**Affiliations:** 1 Departments of Gastrointestinal Surgery, Guilin Medical University, Affiliated Hospital, Guilin, Guangxi 541001, P.R. China; 2 Hepatobiliary Surgery, Guilin Medical University, Affiliated Hospital, Guilin, Guangxi 541001, P.R. China; 3 Pathology, Guilin Medical University, Affiliated Hospital, Guilin, Guangxi 541001, P.R. China

**Keywords:** opioid receptor, small intestine, ischemia-reperfusion injury, protection, signal transduction pathways

## Abstract

Previous studies have demonstrated that (D-Ala2, D-Leu5)-enkephalin (DADLE) protects rats from hepatic ischemia/reperfusion (I/R) injury. In the present study, DADLE was also observed to alleviate IR-induced intestinal epithelial cell injury in rats by inhibiting mitogen-activated protein kinase kinase 7 (MKK7)-c-Jun N-terminal kinase (JNK) pathway signaling. To investigate the protective effect of DADLE on hypoxia/reoxygenation injury in rat intestinal epithelial cells, rat intestinal epithelial cells were treated with different concentrations of DADLE, following which the cell survival rate was determined using a tetrazolium (MTT) colorimetric assay, and apoptosis was determined using flow cytometry. To confirm whether the protective effect of DADLE was due to its effect on MKK7-JNK signaling, the phosphorylation levels of MKK7 and JNK were analyzed using western blot analysis following treatment with different concentrations of DADLE. The results demonstrated that, following treatment with DADLE, the survival rate of the rat intestinal cells subjected to I/R-induced injury increased significantly and the apoptotic rate decreased in a concentration-dependent manner. In addition, the levels of phosphorylated MKK7 and JNK decreased in a concentration-dependent manner following treatment with DADLE. Silencing the gene expression of MKK7 using small interfering RNA prior to DADLE treatment resulted in a reduction in the protective effects of DADLE on the rat intestinal epithelial cells subjected to I/R injury. Collectively, the results of the present study demonstrated that the protective effects of DADLE in I/R injury in rat intestinal cells occurred through inhibition of the MKK7-JNK pathway.

## Introduction

Ischemia/reperfusion (I/R) injury defines a pathological process, in which the ischemia-induced injury of organs or tissues is exacerbated upon reperfusion of the tissue by the blood supply. If I/R injury is not prevented or treated immediately, organ failure and tissue structural damage can occur, which can be life threatening (1). Intestinal tissue is particularly sensitive to ischemia- and hypoxia-induced injury. Intestinal I/R events are of significant concern with respect to clinical conditions, including severe trauma, shock, mesenteric vascular disease, abdominal aortic aneurysm surgery and intestinal transplantation (2–3). Previous studies have demonstrated that intestinal bacterial translocation occurs in ~46.4% of intestinal transplantation recipients, predominantly due to an increase in the permeability of the intestinal wall due to intestinal mucosal barrier damage. As a result, bacteria and their toxins readily pass through the mucosal barrier to cause serious infection or possibly multiple organ dysfunction syndrome (MODS) (4). Therefore, intestinal I/R injury is considered a key initiator in the occurrence and development of MODS and is commonly considered a promoter of MODS (5). Therefore, investigations focussed on elucidating the mechanisms associated with I/R injury and on the prevention of intestinal I/R injury may have important clinical significance.

Since their discovery, opioid peptides and opioid receptors have been a significant area of investigation in the life sciences. Since the first report identifying the involvement of opioids in I/R injury by Schultzsh *et al* (6), an increasing number of studies have demonstrated that opioid receptors and their agonists reduce I/R injury in tissues by affecting various pathways (7,8). Of the three classic opioid receptor groups, *µ*, δ, and κ, (D-Ala2, D-Leu5)-enkephalin (DADLE) is a small molecule δ receptor agonist that was developed and synthesized by Sigma-Aldrich (St. Louis, MO, USA). DADLE has been observed to specifically activate the δ receptor and studies have demonstrated that treatment with DADLE can have a protective effect on I/R injury in heart and brain tissue (9,10). In addition, DADLE has protective effects in I/R injury models of other organs, including the lung, liver and kidney (11–13). However, reports addressing the protective role of DADLE on I/R injury in intestinal tissues remain limited. A previous study also reported that the JNK pathway is important in apoptosis and I/R injury events (14). Therefore, the present study analyzed the JNK pathway to investigate the effect of DADLE on I/R injury in rat intestinal epithelial cells. The results may indicate whether DADLE reduces I/R injury in rat intestinal epithelial cells through the mitogen-activated protein kinase kinase 7 (MKK7) and c-Jun N-terminal kinase (JNK) pathways.

## Materials and methods

### Establishment of an in vitro I/R model in rat intestinal epithelial cells

The present study was approved by the ethics committee of Guilin Medical University (Guilin, China). The CRL-1592 rat small intestinal epithelial cell line (American Type Culture Collection, Rockville, MD, USA) was cultured in Dulbecco's modified Eagle medium (DMEM), supplemented with 10% fetal bovine serum (FBS), 2 mM glutamine, 1% streptomycin and 1% penicillin (all Bao Biological Engineering, Co., Ltd., Dalian, China) in a 37°C CO_2_ incubator. An *in vitro* I/R injury model of intestinal epithelial cells was established by exposing the cells to hypoxia and reoxygenation. For ischemia, the intestinal epithelial cells were cultured in FBS-free DMEM medium in 0.5% O_2_, 5 CO_2_ and 94.5% N_2_ overnight. Reoxygenation of the cells was performed at pre-designated time-points.

### Detection of cell viability

The intestinal epithelial cells (1×10^4^ cells/well) were inoculated into a 96-well plate and were cultured under the ischemic conditions overnight. Different concentrations of DADLE (1, 10, 100 and 1,000 *µ*m) were added to the cells, followed by the reoxygenation treatment for 6 h. Subsequently, 20 *µ*l tetrazolium (MTT; Bao Biological Engineering, Co., Ltd.) solution was added to each well and the cells were cultured for an additional 4 h. Following incubation with MTT, the culture medium was carefully removed, and each well received 150 *µ*l dimethyl sulfoxide. The plate was then placed on a shaker and vortexed at low speed for 10 min. The optical density (OD) atA570 nm of each well was measured using a microplate reader (SpectraMax Plus 384; Molecular Devices, LLC, Sunnyvale, CA, USA).

### Detection of apoptosis

The intestinal epithelial cells (1×10^4^ cells/well) were digested with 0.25% trypsin. Following washing the cells, 100 *µ*l binding buffer and 10 *µ*l fluorescein isothiocyanate (FITC)-labeled annexin-V (20 *µ*g/ml; Bao Biological Engineering, Co., Ltd.) was added to the cells, and the cells were incubated at room temperature in the dark for 30 min. Following incubation, 5 *µ*l propidium iodide (PI; Bao Biological Engineering, Co., Ltd.) was added to each well and the cells were incubated in the dark for 5 min. Following the addition of 400 *µ*l binding buffer to each well, the cells were immediately analyzed using flow cytometry. Cells, which were not treated with annexin-V-FITC and PI were used as negative controls.

### Cell cycle analysis

The cells (1×10^4^ cells/well) were digested using trypsin and collected. The cells were then washed twice with phosphoate-buffered saline (PBS) and the supernatant was discarded. The cells were resuspended in 1 ml 70% pre-chilled ethanol and fixed at 4°C for at least 12 h. The cells were then washed with PBS and centrifuged at 300 × g for 5 min. The cells were washed twice and were then resuspended in 0.5 ml PBS. PI and RNase A (10 mg/ml) were then added to a final concentration of 50 *µ*g/ml, and the cells were incubated in a 37°C water bath for 30 min. Cell cycle analysis was then performed using flow cytometry.

### Western blot analysis

The intestinal epithelial cells (1×10^4^ cells/well) in each group were lysed to extract the total protein (7 M urea, 2 M thiourea, 4& (w/v) CHAPS; 40 mM Tris, 40 mM DTT, 2% phamalyte; pH 3–10). Following determination of the protein concentrations using a bicinchoninic acid method (Nanjing KeyGen Biological Technology Co., Ltd., Nanjing, China), equal quantities of the samples (50 *µ*g) were separated using 10% sodium dodecyl sulfate-polyacrylamide gel electrophoresis (SDS-PAGE). The proteins then were transferred onto a polyvinylidene fluoride (PVDF) membrane (EMD Millipore, Billerica, MA, USA) using a semi-dry method and the membrane was blocked in 5% skim milk at 4°C overnight. Subsequently. the membrane was washed with Tris-buffered saline with Tween 20 (TBST; Sigma-Aldrich), following which the primary antibody was added and incubated at 37°C for 1 h. The following mouse anti-human primary monclonal antibodies (1:500 dilution) were used: Anti-caspase-3 (cat. no. sc-7272), anti-caspase-9 (cat. no. sc-56073), anti-phosphorylated-JNK (cat. no. sc-81502) and anti-JNK (cat. no. sc-7345) (all Santa Cruz Biotechnology, Inc., Dallas, TX, USA). The membrane was washed with TBST, and the appropriate goat anti-mouse secondary antibody (1:1,000 dilution; cat. no. L3032-2; Signalway Antibody, LLC, College Park, MD, USA) was incubated with the membrane at 37°C for 1 h. The membranes were washed with TBST, and the protein bands were developed for 5 min using an autoradiography method (G:BOX Chemi XR5; Syngene, Cambridge, UK). The OD measurements were calculated using Quantity One version 4.6.2 software (Bio-Rad Laboratories, Inc., Hercules, CA, USA). The results are presented as the OD value of the samples / OD value of the internal control.

### small interfering (si)RNA transfection

Serum-free DMEM (50 *µ*l) and 20 pmol of each siRNA (Invitrogen Life Technologies, Carlsbad, CA, USA) were gently mixed. SiMi transfection reagent (1 *µ*l) was diluted in 50 *µ*l serum-free DMEM, mixed gently, and incubated at room temperature for 5 min. The diluted siRNA and SiMi transfection reagent (Shanghai Integrated Biotech Solutions Co., Ltd., Shanghai, China) were then mixed, and 100 *µ*l siRNA/SiMi transfection reagent mixture was added to the appropriate wells of a culture plates containing the cells and culture medium. The cells (1×10^4^ cells/well) were incubated in a CO_2_ incubator at 37°C for 24–48 h.

### RNA extraction and reverse transcriptase-quantitative polymerase chain reaction (RT-qPCR) detection

The total mRNA of the cells in each group were extracted using TRIzol reagent (Invitrogen Life Technologies). Following quantitation, the total mRNA was reverse transcribed into cDNA (FastQuant RT kit; Tiangen Biotech Co., Ltd., Beijing, China), which was used as a template for RTqPCR. Based on the gene sequences in GenBank (http://www.ncbi.nlm.nih.gov/genbank), primers were designed using Primer Premier 6.0 software (Premier Biosoft, Palo Alto, CA, USA). The primer sequences of MKK7 and β-actin were as follows: MKK7, forward 5′-GCCAGACTGGGAAGAAATCTG-3′ and reverse 5′-GGCGGACACACACTCATAAAACAGA-3′ and β-actin forward 5′-CTGGGACGACATGG AGAAAA-3′ and reverse 5′-AAGGAAGGCTGGA AGAGTGC-3′. qPCR amplification was then performed, using SYBR Green PCR Master Mix and QuantStudio 6 (Applied Biosystems Life Technologies, Foster City, CA, USA). The PCR reaction mixture contained: 12.5 *µ*l 2X PCR Master Mix, 2.0 *µ*l cDNA, 1.0 *µ*l forward primer, 1.0 *µ*l reverse primer, and 8.5–25 *µ*l sterilized ionized water. The PCR cycling conditions were as follows: Initial denaturation at 94°C for 5 min, followed by 35 cycles at 94°C for 45 sec, 55–60°C for 45 sec and 72°C for 45 sec, and a final extenstion step at 72°C for 7 min. Following PCR, 5 *µ*l of the amplification product was loaded onto a 1% agarose gel (Thermo Fisher Scientific, Inc., Waltham, MA, USA), containing 0.5 *µ*g/ml ethidium bromide. The DL 1000 Marker molecular standard (Bao Biological Engineering, Co., Ltd.) was used as a reference. Electrophoresis was performed at a voltage of 90 V for 1 h. The bands were visualized and images were captured using an automatic gel imaging system. Images were analyzed using Genetool imaging analysis software (GeneSys version 1.2.5.0; Synoptics Ltd., Cambridge, UK).

### Animal model and sample collection

A total of 40 Sprague-Dawley rats, including 18 females and 22 males, were provided by the Animal Center of Guilin Medical University. The rats weighed between 220 and 280 g and were fasted for 12 h prior to surgery. Anesthesia was performed by an intraperitoneal injection of 20% urethane. Once anesthetized, the right jugular vein was exposed, and an indwelling needle was placed in the vein to systemically administer 2 mg/kg heparin for systemic anti-coagulation. Following removal of abdominal hair, the abdominal cavity was opened, layer by layer, in accordance with the principles of sterile surgery. The small intestine was pushed rightward to expose the aorta and to identify the superior mesenteric artery. The superior mesenteric artery was occluded for 1 h using a vascular clamp, following which the artery was reopened. At 2 h following reopening of the superior mesenteric artery, the rats were sacrificed by cervical dislocation for analysis. As a sham treatment control, the superior mesenteric artery was exposed, but not occluded. In the drug treatment group, DADLE was injected intravenously 10 min prior to the induction of intestinal ischemia. Following sacrifice of the rats, the intestinal segment 10 cm above the cecum was excised. The intestinal tissue was washed with ice-cold saline and dried with filter paper, some samples were immediately stored in liquid nitrogen for subsequent detection of the activities of superoxide dismutase (SOD), malonaldehyde (MDA) and myeloperoxidase (MPO), according to the manufacturer' instructions of the respective kits (Nanjing Jiancheng Bioengineering Institute, Nanjing, China). Whole blood samples (5 ml) were collected from the rats and centrifuged at low temperature, following which the plasma samples were obtained for the detection of diamine oxidase (DAO) by ELISA (Bao Biological Engineering, Co., Ltd.).

### Immunohistochemistry (IHC)

Conventional IHC staining was performed using a streptavidin-peroxidase staining method. The primary antibody was diluted at a ratio of 1:100. A negative control, a blank control and an alternative control were included for comparison. The signals from the stained sections were observed under a light microscope (Axio Scope A2; Zeiss, Oberchoken, Germany). The number of positive cells in a total of 500 cells was determined for each sample. The samples were considered positive if the positively stained cells accounted for >10% of the total cells counted, and samples were considered negative if the positively stained cells accounted for <10% of the total cells counted.

### Statistical methods

The experimental results were analyzed statistically using SPSS 16.0 software (SPSS, Inc., Chicago, IL, USA). Statistical analyses were performed using analysis of variance and χ^2^ tests. Quantitative data are presented as the mean ± standard deviation. P<0.05 was considered to indicate a statistically significant difference.

## Results

### DADLE reverses I/R-induced growth inhibition of intestinal epithelial cells

The I/R-treated intestinal epithelial cells were incubated with different concentrations of DADLE (1, 10, 100 or 1,000 *µ*M) for 24, 28 and 72 h. Cell viability was determined using an MTT assay (Fig. 1). The results demonstrated that following treatment with DADLE, the hypoxia-injured intestinal epithelial cells exhibited increased growth, in a concentration-dependent manner. The increase in growth was most marked in the cells treated with 100 *µ*M DADLE. These results suggested that DADLE reversed the I/R injury-induced growth inhibition of the intestinal epithelial cells.

### DADLE inhibits IR-induced apoptosis in intestinal epithelial cells

The intestinal epithelial cells were subjected to hypoxia for 12 h, at which point the cells were reoxygenated and treated with 100 *µ*M DADLE for 12 h. The levels of apoptosis were then determined using flow cytometry (Fig. 2). The results revealed that apoptosis was observed in 20.6% of the cells in the I/R group, whereas, in the group treated with DADLE, apoptosis occurred in 11.18% of the cells (P<0.01). These results indicated that DADLE had a significant protective effect on I/R injury-induced intestinal epithelial cell apoptosis.

### DADLE reverses I/R-induced cell cycle arrest in intestinal epithelial cells

To investigate whether DADLE affects cell cycle arrest in intestinal epithelial cells induced by I/R injury, cell cycle analysis was performed. Compared with the control group, the cell cycle profile of the intestinal epithelial cells in the I/R group revealed that the cells were arrested in the G0/G1 phase. In the cells treated with DADLE, the cell cycle profile demonstrated that the cells were in the G2/M phases of the cell cycle (Fig. 3). These results suggested that DADLE reversed I/R-induced cell cycle arrest in the intestinal epithelial cells and promoted cell proliferation.

### Effects of DADLE on the I/R-induced expression of apoptosis-associated proteins in intestinal epithelial cells

To investigate the effects of DADLE on the I/R-induced expression of apoptosis-associated proteins in intestinal epithelial cells, the expression levels of caspase family member proteins were determined using western blotting (Fig. 4A and B). The results demonstrated that I/R injury significantly increased the protein expression levels of caspase-3 and caspase-9 in the intestinal epithelial cells, and this increase in the expression of caspase was suppressed following treatment with 100 *µ*M DADLE. These results suggested that the anti-apoptotic effects of DADLE in the presence of I/R injury coincided with the downregulation of caspase family members.

### Effects of DADLE on the protein levels of phosphorylated and total MKK7 and JNK in intestinal epithelial cells subjected to I/R

To investigate the molecular mechanism underlying the protective effects of DADLE against I/R injury in intestinal epithelial cells, the protein expression levels of the MKK7-JNK signal transduction pathway were analyzed using western blotting (Fig. 4C and D). The results revealed that I/R injury significantly increased the protein levels of phosphorylated MKK7 and increased the protein levels of total and phosphorylated JNK. Treatment of the cells with 100 *µ*M DADLE reversed the I/R-induced increase in the phosphorylation of the MKK7 and JNK proteins and reversed the increase in the protein expression of total JNK. Notably, the total quantity of MKK7 protein did not change following treatment with DADLE. These results suggested that DADLE downregulated the phosphorylation of MKK7, thereby protecting the intestinal epithelial cells from I/R injury through the attenuation of JNK signaling.

### Expression of MKK7 in intestinal epithelial cells is silenced by RNA interference

RNA interference technology was used to silence the expression of transcripts within the JNK pathway. Control siRNA and MKK7 siRNA were separately transfected into intestinal epithelial cells. The mRNA and protein expression levels of MKK7 were detected using RT-qPCR and western blotting, respectively. The results demonstrated that, following transfection with 57 nM MKK7 siRNA for 24 h, the mRNA expression of MKK7 mRNA in the intestinal epithelial cells was significantly downregulated. The protein expression of MKK7 also decreased, compared with the control (Fig. 5A and B). These results suggested that MKK7 siRNA transfection effectively silenced the mRNA and protein expression levels of MKK7S.

### MKK7 knockdown reverses the protective effect of DADLE on I/R-injured intestinal epithelial cells

To investigate whether MKK7 knockdown reversed the protective effect of DADLE on I/R-injured intestinal epithelial cells, cell viability was analyzed using an MTT assay and apoptosis was analyzed using flow cytometry. The results revealed that, following MKK7 gene silencing by RNA interference, I/R caused an increase in intestinal epithelial cell apoptosis, leading to a significant decrease in cell survival. Treatment with DADLE did not protect the MKK7-knockdown intestinal cells against I/R-induced apoptosis (Fig. 6). These results suggested that the protective effect of DADLE against I/R injury in intestinal epithelial cells was, at least in part, associated with MKK7.

### Protective effect of DADLE on I/R injury in the rat intestine

To determine the protective effect of DADLE on I/R injury in the rat intestine *in vivo*, an animal model of I/R injury in the rat intestine was established. Following injury, intestinal tissues and whole blood samples were collected and the expression level of DAO in the plasma and the levels of MPO, SOD and MDA in the intestinal tissues were determined (Table I). In addition, intestinal tissue injury and the expression of MKK7 were assessed using IHC (Fig. 7). The results demonstrated that, compared with the control group, the level of DAO in the rat plasma, and the levels of MPO and MDA in the intestinal tissues were significantly decreased. The expression of SOD was significantly higher in the DADLE pre-treated group compared with the control group. In addition, intestinal tissue injury was significantly relieved and the expression of MKK7 was reduced in the DADLE treatment group, compared with the control. Collectively, these results demonstrated that DADLE had a significant protective effect against I/R injury in the rat intestine.

## Discussion

Previous studies have confirmed that the JNK pathway has a close association with I/R injury. A study performed by Uerara *et al* (15) revealed that the JNK signaling pathway is involved in I/R injury in the liver. In a rat myocardial I/R injury model, the AS601245 JNK inhibitor was observed to significantly reduce apoptosis in rat myocardial cells and decrease the area of myocardial infarction (16). Similarly, the SP600125 JNK inhibitor also improved I/R injury in rats following lung transplantation (17), and treatment with the AS601245 JNK inhibitor in a gerbil brain I/R model significantly reduced I/R-induced neuronal apoptosis (18). Using local I/R models, a previous study demonstrated that the activity of JNK in ischemic areas is significantly increased, and treatment with the SP600125 JNK inhibitor inhibits the translocation of B-cell-associated X protein between the cytoplasm and the nucleus, thereby inhibiting neuronal apoptosis and reversing pathological changes (19). MKK4 and MKK7 are two immediate upstream kinases of JNK, and they induce the phosphorylation of JNK at Thr183 and Tyr185 to activate JNK (20). However, these two kinases have functional differences: MKK4 preferentially phosphorylates Tyr185, whereas MKK7 primarily phosphorylates Thr183 (21). The JNK pathway is important in I/R injury, and MKK4 and MKK7 are the only known kinases upstream of JNK. Therefore, inhibition of the phosphorylation of these sites may effectively inhibit JNK activation. In the present study, preliminary experiments revealed that DADLE had a protective effect on rat intestinal I/R injury. Furthermore, it was hypothesized that DADLE reduced intestinal I/R injury through the MKK7-JNK pathway. To confirm this hypothesis, the present study used a cellular hypoxia/reoxygenation model to simulate I/R injury in intestinal cells, and used different concentrations of DADLE to treat the cells following injury. The results of the MTT assay revealed that cell survival increased and apoptosis decreased following treatment with DADLE, in a dose-dependent manner. Western blot analysis was used to detect the protein expression levels of MKK7 and JNK, which demonstrated that as concentrations of DADLE increased, the protien expression levels of MKK7 and JNK decreased, concomitant with a decrease in apoptosis. MKK7 is an upstream molecule within the JNK pathway, which led to the hypothesis that MKK7 was important in the DADLE-mediated protection of intestinal cells subjected to I/R injury. To further confirm the importance of MKK7 in the DADLE-mediated protection of rat intestinal epithelial cells, the gene expression of MKK7 was silenced using siRNA. MKK7 silencing inhibited the protective effects of DADLE on the intestinal cells subjected to I/R injury, which was consistent with the findings from a study by Tang *et al* (22). To confirm whether DADLE had protective effects on intestinal I/R injury *in vivo*, a rat intestine I/R model was used to observe rat intestinal injury following pre-treatment with DADLE. The results of this investigation revealed that DADLE significantly reduced the release of MDA and MPO from the I/R-treated rat intestinal tissues, while the expression of SOD increased and the expression of MKK7 decreased. These results suggested that the I/R injury in the rat intestinal tissues was accompanied by oxidative stress and a reduction in the capacity of the intestinal cells to clear oxygen-based free radicals. Therefore, MKK7 was considered to be a key protein involved in mediating the protective effect of DADLE on intestinal I/R injury. Furthermore, MKK7 may mediate the DADLE-induced alleviation of cellular lipid peroxidation injury, thereby reducing I/R injury in the rat intestine.

Previous studies have demonstrated that the MAPK signal transduction pathways include the extracellular signal-regulated protein kinase (ERK) pathway, the JNK pathway, the p38 pathway and the ERK5 pathway (23). JNK is a cellular enzyme involved in signal transduction, which is associated with cell proliferation, differentiation and apoptosis (24). JNK can mediate apoptosis in various cell types and can contribute to the induction of apoptosis. JNK-mediated apoptosis involves two mechanisms: The first mechanism involves the transcription factor pathway, which occurs through death receptor signaling or mitochondrial-dependent pathways, mediated by the transcriptional regulation of downstream regulatory factors and the expression of apoptosis-associated proteins (25). The second mechanism is the non-transcriptional pathway. During the activation of JNK, a portion of activated JNK remains in the cytoplasm and directly affects the Bcl-2 family members through phosphorylation, regulating their activity and promoting apoptosis through mitochondrial permeabilization (26). The results of the present study suggested that DADLE did not inhibit the protein expression of total MKK7, but inhibited the activation of MKK7. Therefore, it was suggested that DADLE may protect I/R-injured intestinal epithelial cells through the non-transcriptional pathway.

MKK7 is a component of the MAPK signal transduction pathway and is a direct upstream kinase of JNK. MKK7 can activate JNK through the phosphorylation of Thr-183 and Tyr-185 sites within the VIII region of JNK, thereby transducing extracellular stimulation signals into the cell and nucleus to trigger a series of cellular biological responses. Therefore, the inactivation of MKK7 can inhibit the JNK signal transduction pathway, which may be an effective approach for controlling cellular hypoxia injury (27). *In vitro* investigations have revealed that multiple factors, including oxidative stress, bacterial toxins and the inflammatory cytokine TNF-α can lead to the activation of the p38MAPK and JNK signal transduction pathways in intestinal epithelial cells, resulting in the increased expression of caspase-3 and an increase in apoptosis (28–32). In addition, activation of ERK protein can increase the expression of the anti-apoptotic protein Bcl-extra largre, resulting in an anti-apoptotic stimulus (33). *In vivo* animal investigations have reported that JNK and p38 are activated during the I/R injury response, and that pre-treatment with LL-21640-2, to inhibit JNK and p38MAPH, relieves I/R injury in rat intestines. These results suggest that JNK and p38 may act together to promote intestinal epithelial cell apoptosis, thereby aggravating I/R injury in the intestines (34). In addition, the inhibition of p38MAPK alone reduces intestinal epithelial cell apoptosis and improves intestinal barrier function in rats (35), indicating that the MAPK pathway is closely associated with apoptosis. In the present study, the almost complete suppression of the protein expression of MKK7 through MKK7 gene silencing abrogated the protective effect observed following DADLE treatment of the I/R-injured intestinal epithelial cells; however, no reduction in apoptosis was observed. Based on these results, it was hypothesized that I/R-induced cell damage was likely mediated by various pathways and, in addition to the JNK pathway, MAPK-associated proteins were also involved in the regulation of apoptosis. However, the protein components of MAPK signaling are diverse. During the pathological process of intestinal I/R injury, particularly in the early stages, the involvement of JNK, ERK and p38, the activation of MAPK proteins, and the mechanisms underlying the role of activated MAPK proteins in the regulation of I/R-induced apoptosis remain to be elucidated. Future investigations are required to clarify the complex interactions between the MAPK signaling pathways and I/R injury in various tissues.

## Figures and Tables

**Figure 1:** DADLE reverses the I/R-induced growth inhibition of intestinal epithelial cells. Following treatment with different concentrations of DADLE (1, 10, 100 or 1,000 *µ*M) for 24, 48 and 72 h, the viability of the intestinal epithelial cells was determined using an MTT assay. Each independent experimental group was repeated in triplicate. Data are presented as the mean ± standard deviation. ^*^P<0.05. DADLE, (D-Ala2, D-Leu5)-enkephalin; OD, optical density; Model, ischemia/reperfusion.

**Figure 2:** DADLE inhibits ischemia/reperfusion-induced intestinal epithelial cell apoptosis. (A) Detection of intestinal epithelial cell apoptosis using annexin V/PI double staining. (B) Histogram of the percentages of apoptosis in the intestinal epithelial cells. ^*^P<0.01, compared with the model group. Each independent experimental group was repeated in triplicate. Data are presented as the mean ± standard deviation. DADLE, (D-Ala2, D-Leu5)-enkephalin; PI, propidium iodide; FITC, fluorescein isothiocyanate; Model, ischemia/reperfusion.

**Figure 3:** DADLE reverses ischemia/reperfusion-induced cell cycle arrest in intestinal epithelial cells. (A) Cell cycle analysis using flow cytometry. (B) Histogram of the cell cycle distribution of the intestinal epithelial cells, indicating the percentages of cells in the GO/G1 stage. ^*^P<0.01, compared with the control group; and ^#^P<0.05, compared with the model group. Each independent experimental group was repeated in triplicate. Data are presented as the mean ± standard deviation. DADLE, (D-Ala2, D-Leu5)-enkephalin; Model, ischemia/reperfusion.

**Figure 4:** Effects of DADLE on the expression levels of pro-apoptotic proteins caspase-3 and caspase-9 and the expression levels of MKK7 and JNK in intestinal epithelial cells subjected to ischemia/reperfusion. (A) Protein expression levels of caspase-3 and caspase-9 were determined using western blotting. (B) Western blotting results were analyzed using Gel-Pro Analyzer 4.0 software. (C) Protein levels of p- and total MKK7 and JNK were analyzed using western blotting. (D) Western blotting results were analyzed using Gel-Pro Analyzer 4.0 software. ^*^P<0.01, compared with the model group. Each independent experiment was repeated in triplicate. Data are presented as the mean ± standard deviation. DADLE, (D-Ala2, D-Leu5)-enkephalin; Model, ischemia/reperfusion. p-, phosphorylated; MKK, mitogen-activated protein kinase kinase; JNK, c-Jun N-terminal kinase.

**Figure 5:** Expression of MKK7 in intestinal epithelial cells is silenced by RNA interference. (A) Interference efficiency was analyzed using reverse transcription-quantitative polymerase chain reaction following the transfection of 57 nM MKK7 siRNA into intestinal epithelial cells for 24 h. (B) MKK7-knockdown efficiency was further validated by western blotting. MKK, mitogen-activated protein kinase kinase; siRNA, small interfering RNA.

**Figure 6:** MKK7 knockdown reverses the protective effect of DADLE on intestinal epithelial cells following ischemia/reperfusion. (A) Analysis of cell viability using an MTT assay. (B) Analysis of apoptosis using flow cytometry. Each independent experiment was repeated in triplicate. Data are presented as the mean ± standard deviation. ^*^P<0.05, compared with the control group. DADLE, (D-Ala2, D-Leu5)-enkephalin; Model, ischemia/reperfusion; MKK, mitogen-activated protein kinase kinase; OD. optical density.

**Figure 7:** DADLE exerts a protective effect on rat intestinal tissues subjected to ischemia/reperfusion injury by inhibiting the expression of MKK7. Hematoxylin and eosin staining was performed to examine the appearances of the intesstinal tissues in the (A) control group, (B) model group and (C) DADLE-treated group. In the control group, the intestinal mucosal epithelium was intact, and no erosion or ulcers were observed. In the model group, detachment of the mucosa and erosion of the intestinal mucosal epithelium were observed. In the DADLE-treated group, the intestinal mucosal epithelium remained intact. The expression levels of MKK7 in the (D) control group, (E) model group and (F) DADLE-treated group were also examined. In the control group, MKK7 was not expressed at detectable levels. In the model group, marked expression levels of MKK7 were observed. In the DADLE-treatment group, the expression of MKK7 was also observed, although to a lesser extent compared with that in the model group. (Aa–Fa) magnification, ×100; (Ab–Fb) magnification, ×400. DADLE, (D-Ala2, D-Leu5)-enkephalin; Model, ischemia/reperfusion; MKK, mitogen-activated protein kinase kinase. Hematoxylin and eosin staining.

**Table I:** DADLE exerts a protective effect against I/R injury in rat intestinal tissue. Analysis of DAO in rat plasma and MPO, SOD and MDA in rat intestinal tissue.

Group	DAO (*µ*g/*µ*l)	MPO (*µ*g/*µ*l)	SOD (*µ*g/*µ*l)	MDA (*µ*g/*µ*l)
Control	13.43±2.37	0.57±0.16	116.22±13.90	2.49±1.05
I/R	50.64±5.71^a^	1.19±0.21^a^	63.81±15.78^a^	8.74±1.37^a^
I/R+DADLE	27.59±3.99^b^	0.76±0.24^b^	92.91±14.44^b^	3.69±1.28^b^

Each independent experiment was repeated in triplicate. Data are presented as the mean ± standard deviation.

a P<0.05, vs. the control group;

b P<0.05, vs. the I/R group. I/R, ischemia/reperfusion; DADLE, (D-Ala2, D-Leu5)-enkephalin; DAO, diamine oxidase; MPO, myeloperoxidase; SOD, superoxide dismutase; MDA, malonaldehyde.
